# Social impact assessment (SIA) of the Tamale viaduct project in Ghana: Stakeholders management practices, better or worse?

**DOI:** 10.1016/j.heliyon.2023.e14249

**Published:** 2023-03-08

**Authors:** Yakubu A. Zakaria, Tijani Inusah Iddrisu, Barbara K. Arthur

**Affiliations:** a Department of Planning and Land Administration, University for Development Studies, P. O. Box TL1350, Tamale, Ghana; b Department of Sustainable Development Studies, University for Development Studies, P. O. Box TL1350, Tamale, Ghana; c Department of Soil Science, University for Development Studies, P. O. Box TL1350, Tamale, Ghana

**Keywords:** Stakeholder management, Challenges, Strategies, Social impact assessment, Viaduct, Tamale metropolis

## Abstract

Studies have been done in many different fields on how to manage stakeholders, which shows how important it is to put the stakeholder at the center of any program or project. The study looks at the Social Impact Assessment (SIA) of the Tamale viaduct project. The sample size was established using the results of a census. Data was gathered using a key informant interview guide and structured questionnaires using a snowball sampling technique. Out of 128 affected respondents, 120 questionnaires responded to the tools, and three key informant interviews were conducted with significant stakeholders. The analyses show that many communication channels were employed to get in touch with the project's affected stakeholders. Although they were frequently involved, the stakeholders were not allowed to contribute to the decision-making process. The respondents viewed prioritizing the stakeholders, creating a plan for stakeholder involvement, and planning communication as the most effective stakeholder management techniques. Communication problems were cited as a major obstacle to interacting with the stakeholders.

## 1 Introduction

Due to rising concerns about the quality of people's lives and the environment, the Social Impact Assessment (SIA) has become one of the most important parts of starting any project. Because it affects people's health, the growth of industry, urbanization, and technology, as well as their effects on our environment, has for a long time led to a growing concern for better environmental management to improve quality of life [1,2]. How well an assessment of social and environmental impacts works depends on how well and how many people are involved. The same is true for how other projects are evaluated and planned [3].

Ghana's government set up rules and guidelines for environmental control after realizing how important it was to keep the environment in good shape. Under section 2(1) of the Environmental Protection Agency (EPA) Act 1994, the EPA is allowed to make sure that any established Environmental Impact Assessment (EIA) strategies are followed. These strategies help with the planning and implementation of development projects by ensuring consistency with ongoing activities. One of these activities is involving partners in monitoring through EIA support for the right administration [4]. The level of public involvement before, during, and after a project has been started and a big part of how SIA is put together. Stakeholders should be involved and given the chance to give their full input by taking part in all top-level discussions. This is seen as an essential step toward making a SIA that works well and is strong. Getting stakeholders involved has been the subject of many studies, reviews, and criticisms. Local residents, consultants, and businesses should be involved as much as possible at every stage of the process, since their knowledge and experiences will be very important in writing a good SIA report [5].

Stakeholder engagement and public involvement should start on time so that many people can benefit from the project and its problems can be dealt with in a proactive way. Proper stakeholder engagement is important during the planning and execution of projects, so it's important to know how to deal with key stakeholders and communities, especially those who are seen as a threat and have more power over the project [6]. This has been a big problem for many people in charge of projects. When things aren't done right, it could cost the project in the form of disagreements, which could cause the project to be put on hold or even be scrapped. This could also hurt long-term relationships and reputations [7]. Stakeholder participation is a set of steps that make it possible for people who care about the results of a project to help plan and make decisions. They tend to share knowledge and information and work together to make the project more likely to be successful [7].

If the host communities aren't involved in the development of projects, the social, financial, and environmental effects can be bad. It is well acknowledged that the key to any intervention is to engage the local community and other stakeholders in dialogue and foster close relationships with them [6]. Stakeholders are important when it comes to big projects that involve state resources and building infrastructure for people and the local community. People know that some high-profile projects in the fields of roads, oil and gas, transportation, water, etc., have caused a lot of controversy in the public sphere. This is mostly because people think that there wasn't enough planning and project design and that stakeholders weren't consulted enough [8].

As part of its efforts to improve Ghana's social and economic development, the government has set goals to build a transportation system that is integrated, efficient, cost-effective, and sustainable. This will help meet the needs of the public. As a result, this system must encourage growth while reducing poverty [9]. To achieve these goals, the Department of Urban Roads (DUR) aims to cut the average travel time on arterial roads, particularly at crossings, and gradually reduce walking and waiting times for public transportation in low-income neighborhoods and urban centers. Congestion and poor conditions of the existing road network, coupled with a limited number of alternative routes, have resulted in long travel times (queues) and high Vehicle Operating Costs (VOC). In this regard, the construction of the Tamale viaduct seeks to address this bottleneck.

This study aims to clarify stakeholder management practices that occurred in the SIA of the Tamale viaduct project. The research objectives of this paper are 1. to identify the level of stakeholder engagement; 2. to find out the challenges in stakeholder management: and 3. to explore the strategies used for effective stakeholder management. The research results would help us understand the complicated relationships between stakeholders and give project consultants and policymakers ideas for how to make SIA projects more collaborative.

## 2 Literature review

This section's main discussion topics are the conceptual issues and empirical studies connected to stakeholder management techniques in social impact assessment on projects. Precisely, stakeholder engagement challenges involved in stakeholder management and strategies adopted for effective stakeholder management in SIA.

### 2.1 The role of stakeholder engagement in SIA

Stakeholder management is the process of systematically figuring out who the stakeholders are, making plans for them, and putting those plans and strategies into action while working with them [10]. Furthermore, interest in the project is because these stakeholders are impacted by the outcome or involve themselves in the task. Most enterprises, programs, and portfolios will have a broad set of stakeholders with various, sometimes conflicting, interfaces. These individuals, as well as other interest groups, can significantly impact the work's eventual success or failure. Stakeholder management can be defined as a set of approaches for addressing positive benefits while limiting the adverse effects. The four primary steps identified according to Ref. [10] are.

1. Identification of stakeholders
2. Assessment of stakeholder's interest and influence
3. Develop communication management plans
4. Engage and influence stakeholders

Stakeholders will typically include, according to Ref. [11].

1. Individuals and groups performing the work.
2. Individuals and groups affected by the work.
3. Owners, shareholders, and customers.
4. Statutory and regulatory bodies.

In this case, each stakeholder will be marked as having consented to the prospective outcome. Most often, this will take the shape of a lattice that rates affects and interests on a straightforward scale, such as low, medium, or high. Primary stakeholders are sometimes referred to as those who can directly impact the yields or benefits. Stakeholder management becomes more complicated when stakeholders' perspectives, positions, allegiances, and other factors change over time. Because of this, the steps of stakeholder management must be repeated at different times during the project life cycle [10].

Remember the old saying, “No man is an island,” if you want your project to succeed [11]. To answer the “why” question, it's because any project you take on, no matter how big or small, will need help from other people. And it's likely that you would need some kind of help from these stakeholders in terms of their money and time. When good relationships are kept and people are interested, this is called stakeholder management. Effectively communicating with people on a project can make them more likely to stay on the project, and because they may have different levels of interest, they may work on different portfolios [11]. Finally, to any extent, there may be a victory when goals of stakeholders' expectations for the project are met and fulfilled (or, in a perfect world, surpassed) [12].

### 2.2 Challenges involved in stakeholder management in SIA

There are three major sources of Stakeholder Management challenges [13].

1. Unclear Stakeholders–these are stakeholders who cannot espouse their intent enough and are also not truthful about what their interests are in the project;
2. Unidentified Stakeholders–members not noticed early in the project;
3. Unreasonable Stakeholders-these are the stakeholders who do not accept reasonableness and the laws of physics.

The method and control of managing stakeholders must be thoroughly planned out and guided by guiding principles. This involves developing a plan for a company or project based on information (or intelligence) collected through the traditional processes of stakeholder identification, analysis, engagement, stakeholder matrix, and communication. Project because your stakeholders have the power to create or break your project, stakeholder management is crucial [14]. Lack of communication, inadequate resources allocated to the project, modifications to the scope of work, negative news about the scope, and negative community reactions to the job implemented are additional difficulties and vulnerabilities that stakeholders create (cited in: [15]). Again, it is discovered that stakeholders create both challenges and weaknesses when it comes to project implementation [16].

Likewise [17], indicated that substantial sources from all perspectives concurred that including the stakeholders requires a significant time investment, especially if it is to be done well. The extended timeline is prolonged when partners are locked in during more than one point in the ordered survey, as efficient scholars overemphasized. This could be a significant problem for effective surveys given how quickly new enquiries become available. There was disagreement regarding whether the extra time invested results in a progressed item, with some arguing that the time spent with stakeholders was at the very least mostly recovered by avoiding mistakes. Others contend that obtaining the results from the stakeholders' earlier work was more important than include them in the well-designed survey. This time commitment was mentioned as a problem for stakeholders, who typically have other professional or caring responsibilities [18].

In addition to the extra time, lack of resources and preparation limitations can limit stakeholder participation benefits. Many agents lack the knowledge essential to effectively manage such a plan since they are unsure of how to use and interact with stakeholders. Partners who lack a critical background in research may require additional preparation and assistance to commit significantly to the course. Important sources from all angles, particularly effective researchers and those who worked as partners, suggested that both parties should have the necessary foundation and preparation as well as adequate resources to support their respective roles. This would go a long way toward increasing the overall benefit of stakeholder engagement in effective surveys [17].

### 2.3 Strategies for effective stakeholder management in SIA

People's mindset towards strategically managed stakeholders and the stakeholders' perspective in project management encompasses the identification, analysis, communication, decision-making, and all other events associated with managing stakeholders [19]. Identification, communication, analysis, brainstorming, and stakeholder role profile are necessary steps in stakeholder management [20]. The stakeholder management strategy helps to coordinate administrative issues that are often handled separately, such as critical administration, showcasing and human resource administration, organization administration, and social responsibility. The Tonga Climate Resilient Transport Project of the World Bank highlights the value of creating a Stakeholder Engagement Plan (SEP) to enhance and manage stakeholders. The SEP designates an approach that is both technically and culturally appropriate but also calls for discussion and consultation. The SEP's main objective is to promote and enhance decision-making by creating a genuine understanding that includes all parties who will be impacted by the project and various stakeholders. It also makes sure that these parties are given the opportunity to express their feelings and opinions, which will have an impact on project decisions. Keeping track of correspondence and its stakeholders is made easier by the SEP [21].

By setting up meetings where project information (non-technical information) is presented to significant stakeholders, particularly communities, the stakeholders are encouraged to take action. This also gives the group a chance to voice their opinions on what will best serve their interests as stakeholders. Meetings are held to foster relationships with the communities affected by the project [21].

## 3 Study context and methods

### 3.1 Study context

Tamale, traditionally known as Gulkpegu, is Ghana's key transit town to Burkina Faso, Ghana's northern neighbor, and other landlocked countries. It also serves as a major corridor for local and international traffic from the Tema and Takoradi ports to these landlocked countries. Due to its rapid urban growth, Tamale was selected for this study. Traffic in its metropolitan center is backed up by both humans and vehicles; the city has drawn people from far and near, including migrants and immigrants in recent years. It is at the center of Ghana's infrastructural development plan. It serves as the regional capital and the hub for services for Ghana's Northern, Savannah, North-East, Upper-East, and Upper-West regions due to its geographic location and economic importance. The Tamale Metropolitan Assembly (TaMA) is one of Ghana's 261 Metropolitan, Municipal, and District Assemblies and one of the 16 MMDAs in the Northern Region (MMDAs). The Tamale Metropolitan Assembly received a Metropolis designation in 2004 [22].

Tamale is situated between longitude 00.360 and 00.570 East and latitude 9.160 and 9.340 North. East Ganja Municipality is bordered to the north by Savelugu Municipality, the east by Mion District Assembly, the west by Tolon District, and the southwest by Central Gonja District [22]. There are 1,141,708 men and 1,169,235 women living in the Metropolis, which has a population of about 2,310,943 as of the 2021 population and housing census [22]. The proposed project site is within Tamale's Central Business District (CBD). The existing road network comprises the Kumasi–Bolgatanga–Paga Road, the Yendi-Salaga Road, Central Market Road, and Melcom Link (see Fig. 1). Three alignment options of geometric design were produced for the proposed viaduct. The options consisted of two tiers: a flyover with connecting ramps to link the lower tier to the top. In terms of functionality, these were all deemed suitable to serve the purpose of the overhead bridge. In addition to the construction of the viaduct, a total of 10 km lengths (≤10.0 km) of roads were earmarked to be upgraded [9]. This is to ensure all junctions in the screen line are functioning such that they do not impact the overall road network system. The Kumasi-Bolgatanga-Paga Road is a dual-carriageway that forms part of the Economic Community of West African States (ECOWAS) Transnational Road Network, then connects Ghana to Burkina Faso via Paga. The section under consideration is split into two. The first section is from the signalized intersection with Gulkpegu Street, where the Tamale Central Mosque is located, and ends at a ‘T' intersection with Central Market Road. The second section of the road commences from Yendi-Salaga Road, Melcom Link, and the Central Market Road (the Central Market Road is a loop that starts from this intersection and connects back to the Yendi-Salaga Road). This intersection is also signalized [9]; (see Fig. 2).

**Fig. 1:** Project location map. Source: Government of Ghana, 2019.

**Fig. 2:** Bridge layout of Tamale interchange. Source: Government of Ghana, 2019.

### 3.2 Conceptual framework

The concept of triangulation, inside or between methods, refers to the use of different data, theories, and methods to study connected phenomena. This is done to find convergence and confirmation of findings based on both quantitative and qualitative methods (cited in: [23]). Understanding people's opinions and experiences of the social repercussions of the viaduct project is the qualitative objective in this case. The quantitative approach, on the other hand, evaluates the conclusion that there is no appreciable change in the social repercussions associated with the construction of the viaduct. By assessing various but related aspects of social impacts using both methodologies, triangulation seeks to find convergence and validation of both methods' results [24,25]. Fig. 3 depicts the phases that made up this study's mixed methods design.

**Fig. 3:** An illustration of steps involved in the mixed methods design of this study. *Source: Adaptation from* [26].

**Plate 1:** Scaffold Falsework being erected at the fourth three span.

**Plate 2:** Workers removing scaffold falsework from fourth three span (Pm10-Pm13). Source: Field Survey (2022).

### 3.3 Methods

By using questionnaires and key informant interviews to help obtain information, the study used a mixed research methodology. This was crucial because there were so many responders, and they were dispersed throughout the study region. Several techniques and approaches were used to ascertain the level of engagement, challenges, and strategies for effective stakeholder management in SIA on the Tamale Viaduct project, as well as the respondents' knowledge of stakeholder management.

The community and its interpretations of social issues must be considered when evaluating perceptions to guide decision-making and policy implementation. To gain a deeper insight and a better appreciation of people's knowledge, challenges, and methods, it is advantageous to use a case study as a research approach [27]. Affected traders of the project were the main group targeted for the study. Many small and medium-sized businesses at the project location have been relocated due to the viaduct's construction to aid with traffic congestion. The affected people and businesses include banks, taxi drivers, food sellers, mechanics, and store owners, among others. To gather the necessary data, the study took into account each of these individuals.

Stakeholder responses to questionnaires that were specifically designed for this study were gathered and analyzed. The snowball sampling approach was used to choose a sample of the responders [28]. Due to the dispersion of the target population owing to displacement, it was also used to obtain responses from significant external stakeholders participating in the SIA where the chosen project is being carried out. A census was utilized to estimate the approximate number of impacted people in the study population, and the sample size was set so that everyone who was affected was included in the respondents. According to Ref. [9], the reconnaissance survey captured 128 affected persons. Researchers reached out to 120 respondents due to the displacement of affected persons by the project. A census attempts to produce a list of every component in a group and measure one or more of their characteristics [29].

The researchers relied more significantly on source data to create reliable and objective findings. Primary data is essential for a study like this since one gets information directly from the field through the respondents. Key informant interviews (KIIs) were conducted to elicit information from three respondents—the resident consultant of the project, a leader of the affected persons, and an assembly member of the electoral area—as well as closed-ended survey questions that were given directly and indirectly to project-affected people. To compare the data, this research is divided into themes and sub-themes, according to Ref. [30].

The questionnaires were administered in their raw form for quantitative data, which were then edited, coded, and processed for analysis using Microsoft Excel to produce relevant results. For qualitative data, field notes were made via audio recordings, which were thereafter transcribed. The transcripts were subsequently checked and chronologically arranged for thematic analysis within and across cases. This involved a careful review and re-read, which led to finding, examining, and reporting data patterns [31].

## 4 Analytical framework

### 4.1 Kendall's coefficient of concordance

Kendall's coefficient of concordance *(W)* is given by the relation [32]

(1) $$W=\frac{12s}{P^{2}\left(n^{3}-n\right)}-P^{t}$$

and the sum of square statistics (*S)* is given as

(2) $$s=\sum_{i=1}^{n}{\left(R_{i}-R\right)}^{2}$$

where: W is Kendall's coefficient of concordance; P is the number of respondents ranking the challenges; n is the number of quality perceptions; t is the correction factor for tied ranks; while s is the sum of squares statistics over the row sum of ranks (Ri); Ri is row sums of rank; and R is the mean of Ri.

The correction factor for tied ranks (T) is also written as

(3) $$T=\sum_{k-1}^{m}\left(t^{3}-t_{k}\right)$$

where t^3^ is the number of ranks in each the m group of ties.

Therefore, the test of significance of Kendall's coefficient of concordance was done using the chi-square statistics, computed with the equation

(4) $$\chi^{2}=P\left(n-1\right)W$$

There is no consensus among responders regarding the problems, which is the null hypothesis for Kendall's coefficient. If the estimated chi-square exceeds the threshold chi-square, the null hypothesis will be rejected in favor of an alternative one that claims there is agreement in the respondents' rankings of the challenges.

### 4.2 Reliability test

The study estimated the reliability of the research instrument using Cronbach's Alpha. The alpha coefficient (Cα) was calculated to be 0.914, suggesting that the items have relatively high internal consistency, as depicted in Table 1.

**Table 1:** Results of reliability of research instrument using Cronbach's Alpha.

Cronbach's Alpha, Cα	Cα based on standardized items	No. of items
0.914	0.913	19
Valid	120	100
Excluded	0	0
**Total**	**120**	**100**

## 5 Results and discussions

This study discusses the results under four main headings: 1. Characteristics of the affected people; 2. Stakeholder management and extent of engagement; 3. Challenges in stakeholder management; and 4. Strategies for effective stakeholder management.

### 5.1 Background of respondents

This study examined the features of people affected by the Tamale viaduct project. On gender, more females (50.8%) were affected than their male counterparts (49.2%), which suggests dominant female activities in the CBD (see Table 2). The age distribution was almost evenly distributed across the 10-year cohort defined by the study, with the least (11.7%) category being 18–20 years and 31–40 years is the largest (26.7%). This suggests an actively dominated middle-aged workforce within the Metropolis, especially at the project location.

**Table 2:** Background characteristics of respondents.

Variable	Category	Frequency (n = 120)	Percentage (%)
**Gender**	Male	59	49.2
	Female	61	50.8
Total		**120**	**100**
**Age**	18–20 yrs	14	11.7
	21–30 yrs	22	18.3
	31–40 yrs	32	26.7
	41–50 yrs	30	25.0
	51+	22	18.3
Total		**120**	**100**
**Occupation**	Formal Sector	5	4.2
	Trade & Retail	28	23.3
	Services	37	30.8
	Artisan	11	9.2
	Handicraft	21	17.5
	Repair and Maintenance	18	15.0
Total		**120**	**100**
**Education**	Primary	24	20.0
	JHS	25	20.8
	SHS/Vocation	45	37.5
	Tertiary Education	26	21.7
Total		**120**	**100**

According to Ref. [33], the majority of people (15 years and older) are self-employed without employees (60.6%), followed by employees (19.5%), family workers (5.9%), and self-employed (6.9%). The Metropolis' major employer is the private informal sector. The public sector is the second-largest employer, employing 11.3%. Agriculture is only practiced by a small percentage of households (26.1%) within the Metropolis. The highest share of employed people in the Tamale Metropolis (33.0%) is in trade. The survey confirms that a higher proportion of the population is self-employed, particularly in small-scale businesses such as trading goods [33]. This represents slightly over 93.14% of the occupational distribution, dominated by an active informal sector. Only 4.2% of the affected people were formally employed. About one-third (30.8%) were from different service enterprises, such as food vendors, bus conductors, pharmacy operators, and drivers. Other significant categories include trade and retail (23.3%) and handicraft (17.5%), including mechanics, hairdressers, and electricians. Those in the repair and maintenance category were relatively substantial (15%), with the least being artisans. The northern region is noted for arable land, but little can be said of agricultural farming (see Table 2).

On average, all respondents attained different levels of education, ranging from the basic to the tertiary levels. As many as 20% and 20.8% had attained primary and Junior High School (JHS) education, whereas 37.5% were within the level of second cycle education. The relatively educated respondents will likely make consultation and stakeholder engagement issues more effective. This could even be more effective since 21.7% have attained some tertiary education level.

### 5.2 Stakeholder management and extent of engagement in SIA

The concept of SIA is built on the Social Impact Assessment Framework (SIAF), which identifies planning or policy development as one of the most important starting points. SIA is to address both economic loss and social costs from activities that infringe on the free usage of the natural environment. This logic stems from the usual delayed benefits of social and economic projects. More specifically, development projects such as the Tamale Viaduct provide economic benefits and boost to the standard of living, but some adverse effects on the local people often precede this.

Table 3 shows the length of stay of respondents at the project location; 28.5% of the respondents had stayed in the location for 10 years–12 years, while 18.3% had been there for 13 years or more. Only 12.5% of the respondents were found to have stayed there for less than 4 years. This means that most of the respondents on average have been there for at least 5 years, indicating that most respondents would have been fully established in the location, thereby having a normal business cycle. With the project at hand, businesses and routine movements are likely to be hindered, affecting sales, slowing businesses, and even loss of property and business capital.

**Table 3:** Stakeholder management and extent of engagement.

Description	Variable	Frequency (n = 120)	Percentage (%)
**Length of stay at the location of the project site**	0–3 years	15	12.5
	4–6 years	25	20.8
	7–9 years	45	22.5
	10–12 years	31	25.8
	13+ years	22	18.3
Total		**120**	**100**
**Stage of the project life where you contacted**	Feasibility stage	45	37.5
	Implementation stage	19	15.8
	Initiation stage	49	40.8
	Throughout the project life cycle	7	5.8
Total		**120**	**100**
**No. of time of engagement**	Once	31	25.8
	Twice	35	29.2
	Thrice	29	24.2
	Four or more	25	20.8
Total		**120**	**100**
**Receipt/Knowledge of Initial Assessment Report**	No	72	60.0
	Yes	48	40.0
Total		**120**	**100**
**Consideration of Stakeholder Input**	Not at all	56	46.7
	Regularly	13	10.8
	Sometimes	51	42.5
Total		**120**	**100**

The findings also revealed that, in the feasibility and beginning stages of the project, respectively, 37.5% and 40.8% of the respondents were contacted (see Table 3). An indication that the majority were aware of the start of the project. This reflects excellent stakeholder involvement and consultation since most burning issues are supposed to addressed at these stages. The earlier contact with most respondents would have also allowed for in-depth stakeholder inputs and increased project acceptability while reducing divergent stakeholder agitations [34].

Only 29.2% were engaged twice, while 25.8% had a single stakeholder engagement throughout the project. This falls short of the recommended four times stakeholder engagement during a project, as provided by the SIAF. Even though a good number were engaged (i.e., 24.2%) and for four times (i.e. 20.8%), this shows some dissatisfaction since the majority were left out in some of the engagement processes. This lack of adequate engagement could be why 60% were not briefed on the initial assessment report of the project and subsequently poor consideration of stakeholder inputs, as indicated by 46.7% whose inputs were not considered at all. In as much as some inputs from the stakeholders were considered, the poor structuring of such engagements does not show the importance to such inputs (see Table 3).

An interview with a leader of the affected traders revealed the following excerpt on the extent of engagement:

*"It looks like there was a deception about the project because what they told us at the early stage was different from implementation. For instance, at the time of engagement, only opinion leaders were engaged."* (KII with a leader of the affected traders from the Tamale Viaduct project site, 15^th^ April 2022).

According to the leader, not every person in the project's vicinity was contacted. It therefore demonstrates that rather than making sure everyone at the project location was informed of the proposed project to be carried out, quite a few persons were left out of the evaluation.

Contrary to the findings of the study, majority of the respondents were not contacted and involved in the impact assessment during the feasibility and beginning stages of the project [35], they determined that early and widespread stakeholder involvement, as done in the project development procedures, is necessary for social and environmental assessments to be effective. Early stakeholder involvement served to both address some issues before the project started and to assist in producing a thorough report that would be taken into account during project planning and execution.

A contrary account from the consultant engineer for the Tamale viaduct project on the extent of engagement:

*“The affected traders were contacted; let me put it this way, 2018 December was when they were contacted, and the project started in August 2019, so we had a period of about 6/7 months that we were going back and forth with them and the stakeholders. It is not only the people here, but it includes the regional minister, the mayor, opinion leaders and everybody concerned in the assembly”* (KII with a resident consultant of Tamale Viaduct project, 10^th^ March 2022).

From the consultant's perspective, the project was introduced to the residents with a scheme that explained the project's intention. There was a model which included the design and supervision. The design process was for six months, and immediately after the project goes beyond the six months, construction must begin, and once that happens, preceding activities must go on smoothly. However, it took about a year and a half to approve the feasibility report. Contact was made with those who had legal access to the region for their enterprises by formal letters, in-person interactions, and also through an association leader. According to the data gathered, these individuals were engaged twice because the majority of them stated that they had at least two meetings. The Project Management Institute asserted that all project stakeholders needed to be properly informed and educated about the project, listened to, and given opportunities to contribute and provide feedback about the entire process. In contrast, the data mostly refute these assertions [12].

### 5.3 Challenges in stakeholder management in SIA

Table 4 displays the results of the Kendall's coefficient of concordance. The findings show that, with 99% confidence, there is only about 40% agreement among the respondents. The rating indicates that a problem is more severe and more difficult the lower the mean estimate. Out of the eight issues mentioned, the results show that “inadequate identification of stakeholders” is the major barrier. Poor community leader participation, with a mean rank of 4.09, and a lack of communication, with a mean rank of 4.36, came next. The difficulty with the lowest mean rank among the ones offered to the respondents is a lack of coordination, which has a mean score of 4.81. This may be explained by the fact that the majority of respondents and stakeholders were not correctly identified to allow for effective cooperation amongst them. Lack of commitment on parties involved had a mean rank of 4.78being the 6th most important challenge.

**Table 4:** Descriptive statistics on the challenges of stakeholder management.

Challenges	Mean Rank	Rank
Improper identification of stakeholders	3.75	1^st^
Lack of communication	4.36	3^rd^
Lack of coordination	4.81	8^th^
Lack of clear guidelines	4.68	4^th^
Poor participation of community leaders	4.09	2^nd^
Lack of commitment on parties	4.78	6^th^
Poor leadership	4.75	5^th^
Lack of incentives	4.79	7^th^
N	120	
Kendall's W^a^	0.03	
Chi-Square	27.75	
df	7	
Asymp. Sig.	0.00	

A challenge of communication emanates from the study where respondents were not pleased. A statement from the assembly member of Sabonjida, the neighborhood for the viaduct project location, shows an instance of theft during the project life cycle:

*“There was once a theft case at the project site. I reported it to the police. I was not pleased with the way the Consultant handled the case. The thief needed to be punished by the law, but they were only interested in the return of their items. I was unhappy about how the case went”* (KII with assembly member of the project area, 25^th^ February 2022).

There were other communication challenges, as reported by the leader of the affected traders, who revealed the following excerpt:

*There wasn't any communication. They did things independently, and when you even ask questions, the Consultant will tell you that they have been given directives to do their work. On this lane, nobody had been contacted before the project. So, if there are any challenges, we have to question them. As for the engineers, we are with them here, but it's the Consultant who is not from Northern Region. He is there to consult, and maybe it's a private business”* (KII with a leader of the affected traders of the Tamale Viaduct project, 5^th^ March 2022).

As much as respondents were unsatisfied with the level of communication, they still had the intentions of ensuring the project proceeded. Therefore, not allowing issues of theft to go unnoticed.

As explained by Ref. [13], The statistics indicate that respondents disagree and see an unclear stakeholder as a key difficulty, despite the fact that it is one of the major challenges of stakeholder management. This may be the case because those unclear stakeholders who are unable to express their opinions may have others speak for them, particularly those who are affected.

### 5.4 Strategies for effective stakeholder management in SIA

The process of SIA recommends effective stakeholder management as this has the tendency to reduce confrontation among stakeholders while also ensuring some degree of acceptability. Proper identification and involvement of stakeholders ensure acceptability and lead to the achievement of project goals. In assessing strategies for effective stakeholder management, this study used descriptive statistics to determine whether respondents agree with the following strategies relative to effective stakeholder management. With respect to the statement, a mean score above 2.5 denotes relative agreement, while a mean score below 2.5 denotes relative disagreement.

It was found that respondents were almost indifferent (mean = 2.29; SD = 1.103) to the strategy of effective coordination. This means that respondents were not very much in sync with the level of effective coordination throughout the project. This level of response was not so much different from the strategy of understanding relationships (mean = 2.28; SD = 1.117) and that of strong leadership (mean = 2.21; SD = 1.129). However, on the planned communication strategy, there was some common disagreement with that, which shows the low confidence of respondents on that. The strategy of regular meetings was disagreed upon (mean = 2.18; SD = 0.976), indicating the lack of regular meetings among stakeholders. The compensation strategy was also not so different as to the level of disagreement (mean = 2.14; SD = 1.140) which was quite low. This means some compensation was outlined but might have come with strong reservations from affected parties.

Also, even though respondents virtually disagreed (mean = 2.06; SD = 1.132) with the stakeholder identification process, that of stakeholder prioritization was strongly disagreed upon (mean = 1.93; SD = 1.128). This indicates a lack of confidence in the way stakeholders were identified. Poor stakeholder identification and prioritization have a great tendency to affect the outcome of projects. Developing a stakeholder management plan was also strongly disagreed upon (mean = 1.88; SD = 1.081). The fact that all the strategies involving stakeholders are being disagreed upon indicates unsuccessful stakeholder engagement throughout the project (see Table 5).

**Table 5:** Strategies for effective stakeholder management.

Strategies for Effective Stakeholder Management	N	Mean	Std. Deviation
Developing a stakeholder management plan	120	1.88	1.081
Plan Communication	120	2.14	1.056
Strong Leadership	120	2.21	1.129
Regular Meetings	120	2.18	.976
Providing incentives/compensation	120	2.14	1.140
Negotiation	120	2.04	1.088
Understanding relationships	120	2.28	1.117
Effective Coordination	120	2.29	1.103
Stakeholder identification	120	2.06	1.132
Stakeholder Prioritization	120	1.93	1.128
**Valid N (listwise)**	**120**		

Another interesting revelation by this study is the strategies adopted to overcome challenges stemming from the project life cycle. It emerged that different strategies were adopted for all the stakeholders who were affected by the project. We gathered that; the project did not compensate the traders:

*“We were not compensated; we were only given GHS1500 each (approx.205.48 USD at the time of interview) as noise and disturbances fee”* (KII with a leader of the affected traders of the Tamale Viaduct project, 5^th^ March 2022).

The traders were looking at compensation in terms of loss of market structures and the inaccessibility to space for their trading activities.

In terms of negotiation as to how much disturbance fees were to be paid, an excerpt from a Key Informant Interview illustrates that point. Assembly member perspective:

*“There were consultations, and they negotiated about the amount to pay them. But the problem was the story building closer to the public toilet. The owner insisted on his valuer to determine the amount of money due him. He was not ready to allow them to value his property and determine the compensation, which was a major problem for everyone. But I also felt that one person out of about six houses shouldn’t hold the rest to ransom”* (KII with Assemble member of the project area, 25^th^ February 2022).

Resident Consultant perspective:

*“The whole idea of the inconvenience fee was to calm them down, but there was no compensation. For the method of construction, we used scaffolding right to block the whole place (see*Plate 1, Plate 2*). Now they have been removed, so this place looks open. However, before then, one couldn't walk through like this.”* (KII with a resident consultant of the Tamale Viaduct project, 10^th^ March 2022).

It was found that affected people demanded compensation, and there were discussions thereof. However, one disagreeable person in one lane held the others in that lane to ransom (see Plate 1, Plate 2). Some compensation was expected because it was perceived that, a project like this could not have been done without compensation packages, especially when people are likely to lose their livelihoods.

### 5.5 Limitations and future study directives

The study was limited by the time the survey was conducted; i.e., during the project's implementation phase. In hindsight, it would have been prudent to conduct surveys at every phase of the project lifespan; i.e., assessment, implementation, and completion stages, as people are likely to have different perspectives and perceptions at different times. Therefore, for future studies, we recommend that researchers be conscious of collecting data in these phases of the project life cycle.

## 6 Conclusion and policy recommendation

We conclude that, stakeholder management procedures included into the Tamale Viaduct Project's SIA, which frequently worsen the situation for those who are impacted rather than improve it. Every project stakeholder needs to be informed, according to the findings. Owing to the population spread, multiple methods of interaction should be used, such as one-on-one meetings, official letters, and communication through association leaders to reach everyone who cannot be reached through other channels. The study found that in order for the stakeholders to have an impact on certain decisions, SIA needed to meet with them several times and give them access to all discussions. The investigation found that the stakeholders were not properly involved or listened to, and that the choice was occasionally taken into consideration during the process without their awareness.

Therefore, we recommend that, it is advised that effective communication be allowed at all times and at all levels throughout the engagement activities. By learning about the project in-depth and understanding its potential effects, the individuals come to appreciate how important they are to the initiative. Also, a major emphasis should be focused on promptly identifying stakeholders and noting their concerns in order to inform project decisions. To ensure that their solutions are taken into account and integrated into project decisions, those carrying out the project should take the required efforts to engage stakeholders early enough to discuss and negotiate outcomes. This is required to resolve various problems connected to various perspectives without impeding the project's advancement. Finally, stakeholders should have access to and be given a copy of a summary report of the feasibility studies. At all levels of involvement, feedback is really essential. Those stakeholders who couldn't participate in the evaluation may benefit from information provided in a summary report at the conclusion. One strategy to make sure each evaluation aim is met is to adhere to the defined standards for the procedure.

## Author contributions

Conceptualization: Yakubu A. Zakaria; Methodology/Data collection: Yakubu A. Zakaria; Tijani Inusah Iddrisu and Barbara K. Arthur; Data Analysis: Yakubu A. Zakaria, Tijani Inusah Iddrisu and Barbara K. Arthur; Writing (Original Draft Preparation): Yakubu A. Zakaria; Writing (Review & Editing): Yakubu A. Zakaria; Tijani Inusah Iddrisu and Barbara K. Arthur<a name = "Line_manuscript1_138">

## Funding statement

This research did not receive any specific grant from funding agencies in the public, commercial, or not-for-profit sectors.

## Data availability

The data that has been used is confidential.

## Additional information

No additional information is available for this paper.

## Declaration of competing interest

The authors declare no conflict of interest.
